# Strength Abilities and Serve Reception Efficiency of Youth Female Volleyball Players

**DOI:** 10.1155/2022/4328761

**Published:** 2022-06-01

**Authors:** Damian Pawlik, Wioletta Dziubek, Łukasz Rogowski, Artur Struzik, Andrzej Rokita

**Affiliations:** ^1^Department of the Biological and Motor Basis of Sport, Wroclaw University of Health and Sport Sciences, Paderewskiego 35 Avenue, 51-612 Wrocław, Poland; ^2^Department of Physiotherapy, Wroclaw University of Health and Sport Sciences, Paderewskiego 35 Avenue, 51-612 Wrocław, Poland; ^3^Faculty of Health and Physical Culture Sciences, Witelon Collegium State University in Legnica, Sejmowa 5A Street, 59-220 Legnica, Poland; ^4^Department of Biomechanics, Wroclaw University of Health and Sport Sciences, Mickiewicza 58 Street, 51-684 Wrocław, Poland; ^5^Department of Team Sport Games, Wroclaw University of Health and Sport Sciences, Mickiewicza 58 Street, 51-684 Wrocław, Poland

## Abstract

Success in volleyball largely depends on motor abilities, particularly on maximum strength, power, jumping, and speed performance. However, a small number of studies assess the relationship between motor abilities and the effectiveness of volleyball technical skills. Therefore, the aim of the study was to assess the impact of the strength of the upper and lower limbs on the efficiency of serve reception during a 2 vs. 2 game, as well as to evaluate the results of motor measurements in the context of determining the usefulness of current testing procedures. The study involved a carefully chosen group of 12 girls aged 12–13 years (body height: 176.5 ± 4.2 cm, body mass: 58.6 ± 5.1 kg, and training experience: 43 ± 15 months) selected for the Lower Silesian Regional Volleyball Team. The following tests were conducted: handgrip strength with a hand dynamometer, bent-arm hang, 2 kg medicine ball throw, shoulder joint internal rotators (IR) peak torque, standing long jump, spike jump, and countermovement jump. The measurements of the shoulder joint IR peak torque were performed under isometric (at 10°, 35°, and 65° rotation angles) and isokinetic (at 60°/s, 180°/s, and 300°/s) conditions. The efficiency of serve reception was evaluated during a 2 vs. 2 games by using Data Volley statistical software. The strongest positive relationships were observed between the serve reception efficiency and the peak torque and power of the shoulder joint IR, the medicine ball throw distance, and handgrip strength. Jumping variables showed no associations with efficient of serve reception. Consequently, we suggest adding protocols to volleyball training that include strength exercises aimed at developing the IR muscle group. The isokinetic upper limb test should be introduced as a valid tool in selection process. Coaches who do not have access to modern research equipment should use the medicine ball throw test to evaluate strength abilities as an alternative assessment of the serve reception efficiency.

## 1. Introduction

Volleyball requires players to make quick and precise decisions while maintaining highly accurate motor activities. The precision and proper trajectory of the ball that the player hits to a designated place on the court are very important. A player's actions are effective if he or she hits the ball closer to the goal, while efficiency is an additional feature by which a positive result is obtained from the action, regardless of whether the action was intentional. The efficiency index is considered one of the parameters that best explains the team's victory or failure during a game [1].

Palao et al. [2] distinguished two major complexes in volleyball: CI—reception, setting, and attack; CII—block, defense, setting, and counter-attack. The most important activities within these two complexes, which affect the type, form, and consequently the outcome of the play, are the serve and serve reception [3–5]. These two activities have a deciding influence on the subsequent development of play and thus on the result of the game [5–7]. The main goals of the serve are winning a point or making it difficult for the opponent to respond with an effective action. Serve reception is a defensive action, which mainly depends on the type and velocity of the opponent's serve, as well as on the technical and tactical skills of the receiving players [8].

In many sports, success largely depends on the level of skills and motor capabilities and particularly on the ability to develop maximum strength, power, jumping, and speed tasks [5, 9–11]. In volleyball, strength abilities are considered both in terms of the value of maximum muscle contraction and particularly as the relationship between muscle strength and the speed of muscle contraction (force-velocity component) [10, 12]. Serve reception should be performed in a stable position with substantial effort of lower and upper limb movements. A relatively high strength level of the upper and lower limbs may facilitate better ball control by the receiver and a more precise pass to the setter.

According to recent findings, assessments of strength and speed-strength components in competitors from various sports should include measurements of muscle peak torque developed by particular muscle groups in the lower and upper limb joints under isometric or isokinetic conditions, instead of the currently used simple strength field tests [13–15]. In volleyball, the most important tests include a countermovement jump (CMJ) and spike jump with a run-up (SPJ) performed on the force plate to evaluate the power of the lower limbs [16–18].

Current research extensively describes aspects related to the efficiency of the serve, while few studies have attempted to explain the impact of performance on the efficiency of serve reception [19, 20]. Many authors most often use game statistics to determine the merits of this activity [21, 22]. However, no publications have examined the association between the levels of motor abilities with the efficiency of performing particular defensive tasks during a game.

Therefore, the aim of the study was to assess the impact of the strength of the upper and lower limbs on the efficiency of serve reception during a 2 vs. 2 game, as well as to evaluate the results of motor measurements in the context of determining the usefulness of current testing procedures.

## 2. Materials and Methods

### 2.1. Participants

The study involved a carefully selected group of 12 girls aged 12–13 years selected for the Lower Silesian Regional Volleyball Team. Detailed characteristics of the group are presented in Table 1. This team is one of the top three teams in Poland in this age category. Youth volleyball players and their parents were informed about the purpose of the study. Parents provided written permission for their child's participation in the experiment. Before the main tests, each participant was familiarized with the task and performed a practice test. The experiments were performed in the Biomechanical Analysis Laboratory (with PN-EN ISO 9001:2009 certification). The study was reviewed and approved by the Senate Committee on Research Ethics of the Wroclaw University of Health and Sport Sciences, Poland (no. 19/2016), and the procedures complied with the Declaration of Helsinki regarding human experimentation.

Participants were included in study if they were active in competitions and volleyball training. Furthermore, participants must not have currently been experiencing pain in the area of the shoulder girdle; knee or ankle joints and were required to have a current athlete's medical book approved by a sports medicine doctor. Prior to the tests, a dynamic volleyball warm-up was performed, containing only the dynamic exercises, to obtain the highest values of the examined variables. Warm-up includes 2 min trotting, 10 min strength and dynamic exercise (planks, squats, front and side leg swings, trunk twist, hip extension, standing hip rotations, and push-ups), 10 min dynamic warm-up (trotting, arm circles, side shufflers, high knees, butt kicks, lunges, and inchworms), 3 min of coordination ladder exercises, and finishing by 4 min plyometric exercises (alternate leg bounds, 6 m sprint, vertical jump and 6 m sprint, and vertical jump and 6 m sprint with change direction).

### 2.2. Study Design

The following tests were conducted on all players: upper limb tests (muscle peak torque of shoulder joint internal rotators (IR) under isokinetic and isometric conditions, handgrip strength, bent-arm hang, and medicine ball throw), lower limb tests (spike jump, long jump, and countermovement jump with arm swing), and an assessment of the efficiency of serve reception during a game.

### 2.3. Upper Limb Tests

Variables measuring the strength of the upper limbs were assessed using the research tests described below. The handgrip strength of right and left hand was performed with a hand dynamometer (Baseline Hydraulic Hand Dynamometer, White Plains, NY). Next, subjects were required to throw a 2 kg medicine ball and performed the bent-arm hang test [15, 23, 24].

The measurements of the shoulder joint IR peak torque were performed using the Multi Joint 4 isokinetic dynamometer from Biodex Medicine System (Shirley, NY, USA) [25]. Prior to the torque measurements, the seat, dynamometer, and suitable attachment were adjusted to ensure that the tip of the dynamometer became an extension of the axis of rotation of the examined joint. The participant's torso and pelvis were stabilized using straps attached to the chair to eliminate movements in neighboring joints. Next, the internal rotational range of motion of the shoulder joint was established using the control panel. The active internal rotational range of motion was recorded from both shoulders using a standard goniometer technique [26].

The isometric test was performed for the shoulder joint IR at angles of 10°, 35°, and 65°. The measurements for the right and left upper limb (in random order) were performed 3 times for each angle. Participants were required to grip the lever arm while it was positioned in an abduction angle of 90° and elbow flexion angle of 90°, with the forearm in a neutral position. The forearm was in a neutral position in the coronal plane to ensure alignment with the axis of rotation of the dynamometer [27]. This position was considered 0°. Afterwards, verbal instructions were provided, and the test was conducted.

The isokinetic part of torque measurements included the same upper limb position as in an isometric test. The isokinetic test consisted of torque measurements of the shoulder joint IR at the following preset angular velocities: 60°/s, 180°/s, and 300°/s. When the angular velocity was set to 60°/s, participants performed 5 repetitions, while at 180°/s and 300°/s, participants performed 10 and 15 reps, respectively, for a uniform load. A 60-second break was established between subsequent attempts. Participants were required to exert the maximum muscle torque in the shortest possible time for each movement. Based on the registered isokinetic torque values, the power of shoulder joint IR was calculated.

### 2.4. Lower Limb Tests

The height of a spike jump with a run-up was measured using the Vertec Jump Trainer (JUMP USA, Sunnyvale, CA, USA) by tilting the horizontal vanes on the device's extendable arm, which are rotated out of the way by the subject's hand to indicate the height reached [28]. Measurement range of Vertec Jump Trainer was from 170 to 370 cm with an accuracy of 1 cm. The subject stood in front of the training simulator 3 m from the jump mark. The course of motion should reflect the movement of the participant when performing a volleyball attack. Following a run-up, the female athletes performed a spike jump with an arm swing to touch the vane at the highest level possible. The test was performed twice. The greater one of the two results was used for analysis.

Another test was a standing long jump, which was performed in the sports hall on a nonslippery surface. The longer one of the two jumps was measured with an accuracy of 1 cm [23].

CMJ height was measured with using a force plate. The ground reaction forces during jumping were recorded using an ACCUPOWER force plate manufactured by ATMI (Advanced Mechanical Technology Inc., MA, USA) [29]. The sampling frequency for the signal from the platform was set to 240 Hz. Body weight was measured in a standing steady position. On the verbal command “jump,” the subject performed a vertical CMJ with an arm swing. After the jump (100% of one's capabilities), the subject exited the platform and waited for their second jump. The next jump was performed after all subjects had completed the first jump, and the interval did not cause a loss of readiness to attempt the maximum jump. The break between the jumps was approximately 2 minutes. The height of the center of mass was estimated based on the time of flight. Instantaneous peak power in the take-off phase was computed as the product of instantaneous ground reaction forces and the velocity of the general center of body mass. The instantaneous velocity of the general center of body mass in the take-off phase was evaluated based on the integration of the vertical component of the ground reaction forces (reduced by the weight of a participant) with respect to time. The relative peak power was obtained by dividing the peak power by the participant's body mass.

### 2.5. Efficiency of Serve Reception

The volleyball players' game was observed during a tournament for two-person (2 vs. 2) teams. The pairs were created based on a ranking list of all female players, which the team coaches determined based on a subjective evaluation of the game. Coaches considered the following criteria: level of technical skills, level of tactical abilities, and volitional predispositions (determined subjectively—attitude and commitment to training and sports rivalry). Team pairs were selected to ensure that the sum of the ranking number equaled the same value (pairs were created based on the volleyball skills ranking list: 1-12, 2-11, 3-10, 4-9, 5-8, and 6-7). The games were played using “peer-to-peer” system (15 games, 5 games per team). The duration of each game was 14 minutes, and after 7 minutes, the courts were changed. Games were played on a field with the dimensions 18 m × 4.5 m. The height of the net was 215 cm.

Games were recorded using a Sony HD (HDR-CX405) camera. The collected data were subjected to quantitative and qualitative analyses, while the index of efficiency of serve reception of all players was calculated using Data Volley software (Data Project, Italy). The quality of serve reception was assessed on a five-point scale [30]. The serve reception efficiency index was calculated by adding the number of serve receptions of the given type and all serve receptions using the following formula: WE (R) = (R#+R+−R = )/n_dz, where “WE (R)” is an efficiency index, “R#” is a perfect serve reception, “R+” is very good serve reception, “R=” is a serve reception where the opposing team scored a point, and “n_dz” represents the number of players. If a player exhibited a better serve reception, the efficiency index will be closer to 100%.

### 2.6. Statistical Analysis

Statistical analyses were performed using STATISTICA 12.0 software. A basic statistical analysis of the data determined the mean values and standard deviations. The main goal of the statistical analysis was to describe the relationships between the volleyball players' efficiency of serve reception during a 2 vs. 2 game and the investigated motor abilities. Spearman's correlation coefficient *ρ* was determined in the analysis; however, on the basis of the number of participants (*n* = 12), this coefficient was deemed statistically significant when its absolute value was greater than 0.58 (at the significance level *α* = 0.05) or 0.50 (at the significance level *α* = 0.10). Only clear correlations determined from the tested data were considered statistically significant (even if the level *α* = 0.10 is assumed as critical). In the tables below, statistically significant correlations at the level *p* < 0.05 are marked with the symbol (^∗∗^) and at *p* < 0.1 with the symbol (^∗^). The Intraclass Correlation Coefficient was measured for upper limbs on isometric (left ICC = 0.93 and right ICC = 0.95) and isokinetic (left ICC = 0.89 and right ICC = 0.95) tests with confidence interval (95%).

## 3. Results

The strongest statistically significant correlations (*p* < 0.05) were observed between the distance of the medicine ball throw, grip strength of the left hand, isometric peak torque for right shoulder joint IR (65°), isokinetic peak torque for right shoulder joint IR for angular velocities of 60°/s, 180°/s, and 300°/s, and serve reception. Statistically significant relationships (*p* < 0.1) were observed between static peak torque for IR of the left and right shoulder joints at 10° and 35°, isokinetic peak torque for the left shoulder joint IR for angular velocities of 180°/s and 300°/s, and serve reception (Table 2).

The average power (AVGP) of the right shoulder joint IR exhibited significant correlations (*p* < 0.05) with the efficiency of serve reception at all angular velocities (60°/s, 180°/s, and 300°/s), while the power of the left shoulder joint IR exhibited a significant correlation with serve reception at only an angular velocity of 180°/s (Table 3).

## 4. Discussion

The aim of the study was to assess the impact of the strength of the upper and lower limbs on the efficiency of serve reception during a 2 vs. 2 game. First selections for the regional and national teams occur at the age of 12-13. Therefore, this age period is very important for young volleyball players. Currently, studies have evaluated selected motor abilities of female volleyball players [31, 32] or the efficiency of actions during a game with senior players [2, 33]. Anthropometric parameters and motor tests results are decisive factors for the selection of youth national female volleyball teams [34]. However, a small number of works assess the relationship between motor performance and the effectiveness of technical elements in volleyball [35–38]. Katić et al. [35] proved that the mechanisms regulating the force influence the performance of attack, block, and play, while the processes responsible for speed and power have a greater influence on the effectiveness of serve reception. Stamm et al. [36] found that flexibility and speed abilities contributed in 44% to the effectiveness of serve reception. All these works use field-test measurements, while our work includes an extended group of tests with laboratory tests.

The serve reception can have a crucial influence on setting efficiency [39]. All strength tests involving the upper limbs exhibited statistically significant relationships with the efficiency of serve reception, particularly tests in which the IR of the shoulder joint were involved. The achievement of a high strength value may affect the correct positioning of arms at the time of contact with the ball, as well as the accurate reproduction of the technique [40, 41]. Uncontrolled changes in the initiated sequence of movements or in the position of the arms caused by contact with the ball result in a departure from the correct movement pattern and consequently an inaccurate reception or an error. Higher level of strength ability results in greater motor control [42–44]. Thus, athletes with higher levels of upper limb strength will show greater precision and control in the serve reception.

The female player received the serve more efficiently when the value of peak torque of the shoulder joints IR was higher. Higher values for the peak torque and power of the IR within the right shoulder joint generally indicated a more effective serve reception by the player. Significant relationships were observed with the efficiency of serve reception, regardless of the angle or angular velocity at which the torque of IR was evaluated. The vast majority of research describes the results of experienced female players and volleyball players who have recovered from an injury to the upper limb or a comparison between the dominant and the nondominant limb [14, 45–48]. However, no study has investigated volleyball players aged 13 or compared the maximum torque of the upper limbs with the efficiency of actions during a game.

Most volleyball actions (motor activities) are performed in a stable position, but the technique of serve reception itself is based on the movement of the lower limbs, torso, and upper limps towards the ball and following through with a serve reception. Therefore, motor tests in which the isokinetic element occurs are more strongly correlated with technique and consequently with the result of the action performed. On the basis of the results of the assessment of strength abilities, tests that evaluate the peak torque of the shoulder joint IR under isokinetic conditions at high angular velocities of 180°/s and 300°/s using modern research equipment appear to be more reasonable than tests performed under isometric conditions. Coaches who do not have access to modern research equipment should use the medicine ball throw to measure strength as an alternative assessment of the serve reception efficiency [35].

Lower limb tests showed no associations with efficient of serve reception. Wrong chosen strength tests, which do not reflect the specifics of the game, may provide information opposite to the anticipated results. Katić et al. [35] noticed relationship between lower limb movement and effectiveness of serve reception. Tests based on the measurement of movement speed or lower limb power may be more appropriative for the displacement to the incoming ball than for the serve reception effect itself (when a quasistatic position is performed). Therefore, it is worth adding tests based on the isometric torque measurement, which is responsible for stabilizing the position during serve reception. The vertical jump height and power did not significantly affect the efficiency of the serve reception. When analyzing the technique of serve reception, the athlete should assume a stable position with lower limb flexion, undergoing a slight extension at the time of contact with the ball. Therefore, a test should be applied that is more similar in terms of the specificity of serve reception. To identify the relationship between the strength of the lower limbs and the efficiency of serve reception the test based on the isometric effort should be used, rather than a jumping ability test.

Upper body strength is identified as one of the most important factors in differentiating between players of the most and least successful teams [49]. In the present study, we attempted to assess the strength abilities of upper and lower limbs with the efficiency of serve reception. Currently, the efficiency of volleyball technique skills was mostly evaluated only by game statistics or in isolated game fragments. There are insufficient studies about the relationships between serve reception during the game and motor ability test results. While performing isolated movement tasks, the player may perform them with high efficiency but can still commit numerous errors during the game.

Our study has some limitations. The studied athletes were youth female volleyball players; therefore, obtained relationships should not be related to the elderly and male groups. The studied group considered only 12 participants, but it should be taken to account that it was a selected group of female volleyball players with the highest performance level at this age.

## 5. Conclusions

Among the many field and laboratory tests used in this study, it has been shown that IR isokinetic tests have the strongest relationship with the effectiveness of serve reception. Therefore, the IR muscle group has a significant role in successful serve reception. Consequently, we suggest adding protocols to volleyball training that include strength exercises aimed at developing this muscle group. Our research suggests that if possible, the isokinetic upper limbs test should be introduced as a valid tool for selecting female players for representative groups.

## Figures and Tables

**Table 1:** Characteristics of the study group.

Group (*n* = 12)	Body height (cm)	Body mass (kg)	BMI (kg/m^2^)	Training experience (month)
Mean ± SD	176.5 ± 4.2	58.6 ± 5.1	18.8 ± 1.3	43 ± 15.1

**Table 2:** Strength abilities of 13-year-old girls selected for the Lower Silesian Regional Volleyball Team with correlation coefficients with the serve reception.

Variable		Mean ± SD	Confidence interval		Serve reception
			-1.96 SD	1.96 SD	
Handgrip strength (kG)	R	27.3 ± 3.1	25.3	29.3	0.34
	L	27.6 ± 3.4	25.4	29.7	0.64^∗∗^

Isometric peak torque at a specific angle (Nm)	L 65°	19.6 ± 6.0	15.8	23.4	0.4
	L 35°	19.7 ± 5.1	16.5	22.9	0.57^∗^
	L 10°	19.6 ± 5.1	16.3	22.8	0.57^∗^
	R 65°	22.7 ± 5.9	18.9	26.4	0.67^∗∗^
	R 35°	23.0 ± 5.4	16.5	22.9	0.54^∗^
	R 10°	21.8 ± 5.5	16.3	22.8	0.54^∗^

Isokinetic peak torque of IR at a specified angular velocity (Nm)	L 60°/s	19.9 ± 3.8	17.5	22.3	0.34
	L 180°/s	19.8 ± 3.7	17.4	22.1	0.53^∗^
	L 300°/s	23.1 ± 5.3	19.7	26.5	0.54^∗^
	R 60°/s	20.1 ± 4.7	17.2	23.1	0.71^∗∗^
	R 180°/s	18.6 ± 4.4	15.8	21.4	0.72^∗∗^
	R 300°/s	22.7 ± 5.1	19.4	25.9	0.70^∗∗^

Simple field tests (ICSPFT)	Distance the medicine ball was thrown (m)	8.0 ± 1.3	7.2	8.8	0.59^∗∗^
	Bent-arm hang time (s)	29.7 ± 6.9	25.3	34.1	-0.50^∗^
	Standing long jump (cm)	193 ± 9	187	199	-0.29

Jump tests	SPJ reach height (cm)	270 ± 12	262	278	0.08
	CMJ height (cm)	30.5 ± 5.2	27.6	33.8	-0.05
	CMJ peak power (W/kg)	44.5 ± 6.2	41.1	48.4	-0.21

R: right side; L: left side; ICSPFT: International Committee on the Standardization of Physical Fitness Test; ^∗^significant at *p* < 0.1; ^∗∗^significant at *p* < 0.05.

**Table 3:** Average power of the internal rotation of the shoulder joint under isokinetic conditions and the correlation coefficient with the serve reception.

Average power	Mean ± SD (W)	Confidence interval		Serve reception
		-1.96 SD	1.96 SD	
AVGP L IR 60°/s	12.7 ± 2.6	11.0	14.3	0.37
AVGP L IR 180°/s	20.6 ± 4.4	17.9	23.4	0.54^∗^
AVGP L IR 300°/s	21.1 ± 6.3	17.1	25.1	0.45
AVGP R IR 60°/s	13.5 ± 3.5	11.2	15.7	0.77^∗∗^
AVGP R IR 180°/s	21 ± 6.6	16.9	25.2	0.89^∗∗^
AVGP R IR 300°/s	21.5 ± 6.2	17.6	25.4	0.90^∗∗^

^∗^Significant at *p* < 0.1; ^∗∗^significant at *p* < 0.05; R: right side; L: left side; IR: internal rotation.

## Data Availability

The data used to support the findings of this study are available from the corresponding author upon request.
